# Mutational Screening of Skeletal Genes in 14 Chinese Children with Osteogenesis Imperfecta Using Targeted Sequencing

**DOI:** 10.1155/2022/5068523

**Published:** 2022-05-19

**Authors:** Wei Tan, Yuelun Ji, Yuepeng Qian, Yongchang Lin, Ruolian Ye, Weiping Wu, Yibin Li, Yongjian Sun, Jianyin Pan

**Affiliations:** ^1^Department of Pediatric Orthopedic, Center for Orthopedic Surgery, The Third Affiliated Hospital of Southern Medical University, Guangzhou 510515, China; ^2^Department of Joint Surgery, Center for Orthopedic Surgery, The Third Affiliated Hospital of Southern Medical University, Guangzhou 510515, China

## Abstract

**Background:**

As a heterogeneous hereditary connective tissue disorder, osteogenesis imperfecta (OI) is clinically characterized by increased fracture susceptibility. Analysis of genetic pathogenic variants in patients with OI provides a basis for genetic counseling and prenatal diagnosis.

**Methods:**

In this study, 14 diagnosed OI patients from sporadic Chinese families were enrolled to be screened for potential mutations from these patients by next-generation sequencing technology.

**Results:**

34 different variants were identified. 18 variants were from 4 OI-related genes including *COL1A1*, *COL1A2*, *P3H1*, and *WNT1*, and 10 variants are novel. Most OI patients (11 out of 14, 78%) harbor variants in type I collagen genes.

**Conclusions:**

Our results support previously established estimates of the distribution and prevalence of OI mutations and highlight both phenotype and genetic heterogeneity among and within families. We report several novel variants of OI, which expands the clinical spectrum of OI. In summary, our data provides disease-causing genes information for genetic counseling towards OI patients and families and also provides a reference for clinicians in the diagnosis of OI, also in prenatal diagnosis of this disease.

## 1. Introduction

Osteogenesis imperfecta (OI), also known as brittle bone disease, comprises a class of connective tissue disorders characterized by increased bone fragility and vulnerability to fracture due to minor trauma. Other features include brittle teeth, low bone mass, hearing loss, and blue sclera. The incidence of OI was estimated to be 6 to 7 per 100,000 people worldwide [1]. OI is clinically and genetically heterogeneous and historically had various other names. The name OI dates back to at least 1895, and the current four-type system with Sillence began in 1979 [2]. Using clinical, radiographic, and genetic criteria, OI individuals were categorized into four types: type I (mild OI with blue sclera, Mendelian Inheritance in Man (MIM 166200)), type II (pre- or perinatal lethal, MIM 166210), type III (severe deforming, MIM 259420), and type IV (intermediated severity, MIM 166220) in 1979 [3]. However, the correlation between specific genetic defects and clinical manifestations is confused due to the apparent overlap between clinical manifestations and disease severity. Therefore, a new classification system was proposed based on the specific genetic defects that cause the disease [4]. The new revision of classification types 1-4 is closely related to Sillence's previous I-IV classification system. It is mainly based on specific phenotypic characteristics and genetic findings describing other OI types (V and higher). There are currently 23 distinct OI types according to the affected genes according to the Online Mendelian Inheritance in Man (OMIM) resource (https://omim.org). It is established that 90% of OI was caused by variants in the two collagen coding genes (*COL1A2* and *COL1A1*), which cause a lack of type I collagen [5]. These genetic defects are often inherited from a person's parent in an autosomal dominant manner or occur via a de novo mutation. Currently, more and more pathogenic genes have been discovered, which further facilitate OI classification. Variants of *CRTAP* (MIM 605497) and *SERPINF1* (MIM 172860) may be the cause of type VII and VI OI, respectively [6, 7]. The remaining types are usually associated with mutations in some autosomal recessive genes, such as *P3H1* (MIM 610339) [8], *WNT1* (MIM 164820) [9], and *TENT5A* (MIM 611357) [10]. The genetic classification incorporated a new type for each defective mutation. In total, OI is considered to be a spectrum with considerable phenotype overlap between the subtypes. The application of next-generation sequencing technologies (NGS), such as targeted sequencing, whole exome (WES), or whole genome sequencing (WGS), has greatly improved the diagnosis and classification of OI. In particular, targeted sequencing of candidate genes is considered as a cost-effective strategy for the clinical diagnosis of heterogeneous disorders [11]. A recent study reported that targeted sequencing has been applied to prenatal diagnosis of skeletal dysplasia [12].

Considering the increasing popularity of molecular diagnosis during OI classification, we assembled a cohort of 14 OI patients of Chinese ethnicity and investigated their mutation spectrum using a targeted skeletal gene panel. Other than known variants, we identified novel variants associated with OI and revealed the genotype-phenotype relationships.

## 2. Methods

### 2.1. Patients

There were 14 unrelated probands with OI recruited at The Third Affiliated Hospital of Southern Medical University, Guangdong, China, in this project. After obtaining appropriate informed consent from participants and/or legal guardians, the whole blood samples were collected from the affected individuals. All affected individuals including the probands and their family members were of Chinese Han ethnicity. The complete pedigree information for the individuals is summarized in Figure 1. The details of the medical history, phenotype features, and physical examination were obtained and summarized in Table 1. This study was approved by the Institutional Review Board of the Third Affiliated Hospital of Southern Medical University.

### 2.2. Targeted Sequencing and Variant Identification

Due to the clinical and genetic heterogeneity of OI, targeted sequencing was performed on all 14 patients to identify potential variants. Briefly speaking, genomic DNA was extracted from the peripheral blood of patients, using a customized array (NimbleGen, Roche Madison, USA) to capture the whole exons and flanking intronic sequences (±10 bp) from 225 genes known to be associated with inherited skeletal disorders and then followed by high-throughput sequencing on Illumina HiSeq 2000 platform with 150 bp paired-end reads (supplementary Table S1). Bioinformatics analysis was performed using public software and independently developed pipelines. In bioinformatics analysis, all cleaned data after trimming were aligned against human reference genome build hg19 using Burrows-Wheeler Alignment (BWA) tool. The mean depths was 150x across all patients. With the integration of customized databases, SNP and Indels were then discovered by HaplotypeCaller module of the Genome Analysis Toolkit (GATK) and annotated by ANNOVAR. Analysis was restricted to coding and flanking intronic regions which generally ensure good data coverage. Variants with minor allele frequency (MAF) greater than 1% in any of the Exome Aggregation Consortium (ExAC), the Genome Aggregation Database (gnomAD), NHLBI GO Exome Sequencing Project (ESP6500) databases, and 1000 genome project were excluded from subsequent analysis. Then, filtering and prioritizing were performed to look into potentially deleterious variants, including missense, nonsense, indel, frameshift, and variants affecting splicing, for variant interpretation and classification according to American College of Medical Genetics (ACMG) guidelines.

Fragments covering the mutation sites of the relevant genes were amplified by PCR followed by Sanger sequencing to confirm identified mutations of interest. According to the manufacturer's instructions of Premix Taq™ Hot Start Version/TaKaRa LA Taq® with GC Buffer (Takara, Osaka, Japan), PCR amplification was performed under the following conditions: 1 cycle of initial denaturation at 95°C for 2 min and 35 cycles of 95°C for 30 s, 60°C for 30 s, 72°C for 30 s, and 5 min at 72°C. Using an ABI 3730 DNA Analyzer with BigDye™ Terminator Cycle Sequencing Kit (Applied Biosystems, Foster, CA, USA), polymerase chain reaction (PCR) fragments were purified and further sequenced.

## 3. Results

Fourteen clinically and radiologically confirmed patients with OI were selected for this study. Out of them, 9 were males and the remaining 5 were females. Most of them were children, and the average age was 7 years old. All the patients were type III except patient 11. Blue sclera is an important clinical characteristic of OI patients and was observed in 13 patients in our cohort. 10 patients suffered tooth agenesis, and almost all patients (13 in 14) have fracture history. The number of fractures in these patients ranged from 0 to 8. Out of 34 heterozygous variations in total identified, 18 polymorphisms in 4 OI-related genes including *COL1A1*, *COL1A2*, *P3H1*, and *WNT1* and the remaining 16 were in other genes (Figure 2).

The 18 polymorphisms in the 4 OI-related genes were shown in Table 2. 10 variants are novel. 3 mutations are localized within the triple helix repeat of the *COL1A1* gene, 2 in *COL1A2* gene, and 1 in *P3H1* gene. All mutations of *WNT1* gene are novel. Four probands carried splicing variants, including three from *COL1A1* (c.2451+1G > A, c.1821+1delG, and c.693+5G > A) and one from *WNT1* (c.104+1G > A). These four splicing variants were closely related with mild to moderate phenotype features predominantly characterized by short stature and recurrent fractures. Three probands had frameshift mutations, including two from *COL1A1* (p.G1046Vfs∗62 and p.A606Cfs∗27) and one from *WNT1* (p.R73Tfs∗82). One proband carried null mutation in *P3H1* (p.R210X), and the rest were nonsynonymous mutations.

Consistent with the previous reports, *COL1A2* and *COL1A1* were the two most frequently mutated genes (11 out of 14 patients). Locations of variants in *COL1A2* and *COL1A1* in individuals were shown in Figure 3. 7 probands had a *COL1A1* variant. Three variants including c.1721G > A, c.1816_1817del, and c.2069C > T were novel, and the rest four had been reported previously, which include c.2451+1G > A, c.2443G > A, c.1821+1delG, and c.3135delT [13–16]. 5 probands had a *COL1A2* variant, out of which three variants have been reported in previous studies, including c.1801G > A in patient 7, c.693+5G > A in patient 9 [17], and c.964G > A in patient 10 [18]. The splicing variant in patient 9 occurred at a highly conserved site. With respect to *P3H1*, there was a previously reported variation (c.628C > T) [19] and a novel compound heterozygote variant (c.1703G > A). Four novel compound heterozygote variants were detected in the *WNT1* gene, including two nonsynonymous mutations, one splicing variant, and one frameshift variant.

In this report, we present 4 OI probands with substitutions of glycine residue including p.G815S from *COL1A1* and p.G601S, p.G391V, and p.G322S from *COL1A2*. The phenotypes of these probands are consistent with the previous reports that these variants of substitutions are associated with severe OI. For example, patient 5 suffered fracture of left tibia 20 days after birth and fractured right femoral shaft 2 months later. His mother carried this mutation and presented excess fractures. However, the proband with OI may be significantly affected clinically, whereas family members with the same mutation may have no obvious symptoms (patient 6 and her father), demonstrating that the clinical manifestations vary substantially within families with different types of genetic variants.

Additionally, we also found 16 variations in 14 other genes, as shown in Table 3. There were two mutation sites in *RPGRIP1L* (c.1960G > A and c.3272G > A) in patient 14. The protein encoded by *RPGRIP1L* localizes to the basal body-centrosome complex in ciliated cells and takes part in Hedgehog and organelle biogenesis and maintenance pathways. Defects in RPGRIP1L are a cause of Meckel syndrome type 5 (MKS5 and MIM 611561) and Joubert syndrome type 7 (JBTS7, MIM 611560) [20]. Our results suggested that *RPGRIP1L* mutation may be related to OI, which is worthy of further investigation.

## 4. Discussion

OI is an inherited connective tissue disorder with a wide genotypic and phenotypic spectrum and up to 23 subtypes. Mutations in type I collagen or proteins involved in posttranslational modification of type I collagen are the most common cause of OI. Type I collagen containing two *α*1 and one *α*2 chains is a heterotrimeric fibrillar collagen, and *α*1 and *α*2 chains are encoded by *COL1A1* and *COL1A2*, respectively. Genetic defects include reducing the amount of type 1 collagen (quantitative defects) or affecting its structure (qualitative defects), resulting in a milder phenotype to more severe phenotype [21]. The remaining cases were caused by genetic defects in genes involved in the posttranslational modification and intracellular trafficking of type 1 collagen or genes related to osteoblast differentiation and function. In our study, 11 out of 14 patients exhibited mutation in *COL1A1* or *COL1A2*, accounting for 78% of our cohort. There is no hotspot mutation identified in *COL1A1* and *COL1A2* genes.

Other than *COL1A1* and *COL1A2* genes, mutations in *P3H1* and *WNT1* were found in our OI patients. It is known that cartilage-associated protein (encoded by *CRTAP*), cyclophilin B (encoded by *PPIB*), and prolyl 3-hydroxylase 1(encoded by *P3H1*) form a collagen posttranslational modification complex in a 1 : 1 : 1 ratio on the endoplasmic reticulum and regulate collagen function [8]. The null mutation in *P3H1* would result in a protein decrease or absence, leading to the collapse of the complex [8, 22]. The defective structural collagen exhibits a delay in the collagen helix folding and exposes the constituent chains to lysyl hydroxylase and prolyl 4-hydroxylase for a longer period of time, leading to overmodification of the chain [8]. The truncation of *P3H1* gene has been previously reported in OI individuals. In addition, we reported a novel missense variant c.1703G > A, which is the first one ever reported to the best of our knowledge. This missense variant was predicted to be a disease causing by Sift [23] and Polyphen-2 [24].

The *WNT1* encodes a ligand for the WNT signalling pathway, which acts as a primary regulator in bone formation. Wnt1 promotes bone formation by binding to the LRP5-FZD receptor complex and activating the canonical WNT signalling pathway for promoting bone formation. Loss-of-function mutations in *WNT1* result severe OI, severe skeletal abnormalities, white sclerae, or possible neurological defects [25]. Herein, we report four autosomal recessive (AR) forms of *WNT1* variants and two are likely pathogenic. More than 3200 variants have been observed across *COL1A1*, *COL1A2*, *P3H1*, and *WNT1* genes (http://www.le.ac.uk/ge/collagen/).

The type I collagen genes are also associated with other genetic bone diseases including Caffey disease [26], arthrochalasia Ehlers-Danlos syndrome (aEDS) [27–29], cardiac valvular EDS (cvEDS), and OI/EDS disease [30, 31]. The core phenotype is closely related to the location of deleterious defects. Mutations near the N-terminal peptide, which links the N-propeptide to the triple helical domain of collagen, are often associated with aEDS or OI/EDS [32]. Clinical symptoms of OI and OI/EDS overlap. Given the clinical and genetic heterozygosity of these disease, their diagnosis and treatment are always challenging. Hence, detailed clinical characterization of rare diseases is extremely important. In our study, mutations in type I collagen gene cluster in collagen *α* chain are far from the N-terminal peptide. The patient's clinical symptoms did not show increased laxity of the ligaments and skin.

In addition to variations in 4 OI-related genes, our study also identified novel mutations in 14 other genes, such as 2 heterozygous mutations in *RPGRIP1L*. Whether these variants are OI causing or not is worthy of further investigation. Our data support that the autosomal dominant (AD) forms are most prevalent in our Chinese OI population. These results highlight the importance of genetic analysis in autosomal dominant disease including OI, which can significantly reduce the risk of this serious disease. 6 probands were AR forms of OI. Previous studies have reported that approximately 10-20% of germline pathogenic mutations may alter mRNA splicing. There were four splicing mutations found in our analysis. In one of these cases, no pathogenic variants were identified in known OI genes, making them suitable for WGS or WES to identify novel underlying genetic defects of OI.

In summary, our study provides an estimate of the prevalence and the distribution of OI mutations and further highlight both phenotypic and genetic heterogeneity among and within families. The technological improvements and decreasing cost will make NGS approaches an effective first-tier screening method, and the targeted sequencing of interested gene panels has become part of routine clinical genetic practice for the diagnosis of heterogeneous disorders [33]. However, our study was limited to a single center and was retrospective. A larger number of phenotype-genotype correlative studies are required in order to provide better insights into OI.

## Figures and Tables

**Figure 1:** Pedigrees of the individuals described. The black part of Figure 1 represented probands with osteogenesis imperfecta.

**Figure 2:** Summary of variants identified in the study.

**Figure 3:** Location of mutations in *COL1A1* and *COL1A2*. (a) Schematic diagrams indicated the mutation above the *COL1A1* and collagen triple helix repeat domain of the COL1A1 proteins (NP_000079.2). (b) Schematic diagrams indicated the mutation above the *COL1A2* and collagen triple helix repeat domain of the COL1A2 proteins (NP_000080.2).

**Table 1:** Clinical features of the 14 OI patients.

Patient ID	Gender	Age (y)	Blue sclera	Tooth agenesis	Fracture (T)	Contractures	Hearing loss
1	Male	13.8	Yes	No	7	No	No
2	Male	11.1	Yes	No	3	No	No
3	Male	9.3	Yes	Yes	7	No	No
4	Female	3.6	Yes	Yes	2	No	No
5	Male	2.5	Yes	Yes	1	No	No
6	Female	0.75	Yes	No	0	No	No
7	Male	15	No	Yes	5	No	No
8	Female	14.8	Yes	Yes	8	No	No
9	Male	7	Yes	Yes	3	No	No
10	Male	0.6	Yes	Yes	3	No	No
11	Male	10.9	Yes	Yes	3	No	No
12	Female	8.7	Yes	Yes	3	No	No
13	Male	2.75	Yes	No	7	No	No
14	Female	5	Yes	Yes	2	No	No

M: male; F: female; y: year; T: times.

**Table 2:** Variations in 4 OI-related genes.

Patient ID	GENE	Inheritance	Nucleotide variant	Predicted consequence	Zygosity	ACMG	Paternal/maternal
1	*COL1A1*	AD	c.2451+1G > A	Splicing	Het	p	De novo
1	*COL1A1*	AD	c.1721G > A	p.R574H	Het	VUS	Maternal
2	*COL1A1*	AD	c.3135delT	p.G1046Vfs∗62	Het	P	Paternal
3	*COL1A1*	AD	c.1816_1817del	p.A606Cfs∗27	Het	P	De novo
4	*COL1A1*	AD	c.2069C > T	p.P690L	Het	VUS	Maternal
5	*COL1A1*	AD	c.2443G > A	p.G815S	Het	P	Maternal
6	*COL1A1*	AD	c.1821+1delG	Splicing	Het	LP	Paternal
7	*COL1A2*	AD	c.1801G > A	p.G601S	Het	LP	Maternal
8	*COL1A2*	AD	c.1172G > T	p.G391V	Het	VUS	NA
9	*COL1A2*	AD	c.693+5G > A	Splicing	Het	LP	De novo
10	*COL1A2*	AD	c.964G > A	p.G322S	Het	LP	Maternal
11	*COL1A2*	AD	c.746 T > C	p.I249T	Het	VUS	Paternal
12	*P3H1*	AR	c.1703G > A	p.C568Y	Het	VUS	Maternal
12	*P3H1*	AR	c.628C > T	p.R210X	Het	P	Paternal
13	*WNT1*	AR	c.216dupA	p.R73Tfs∗82	Het	LP	Maternal
13	*WNT1*	AR	c.371C > T	p.T124M	Het	VUS	Paternal
14	*WNT1*	AR	c.104+1G > A	Splicing	Het	LP	Maternal
14	*WNT1*	AR	c.501G > A	p.W167C	Het	VUS	Paternal

AD: autosomal dominant inheritance; AR: autosomal recessive inheritance; P: pathogenic; LP: likely pathogenic; VUS: uncertain; NA: parent samples were not available for the analysis.

**Table 3:** Variations in other genes.

Patient ID	GENE	Inheritance	Nucleotide variant	Predicted consequence	Zygosity	ACMG pathogenic	Paternal/maternal
1	*SLC34A1*	AR/AD	c.1322A > G	p.Y441C	Het	VUS	Paternal
1	*LRSAM1*	AR/AD	c.1367C > T	p.A456V	Het	VUS	Paternal
3	*ACVR1*	AD	c.454C > T	p.R152C	Het	VUS	Maternal
4	*ACAN*	AR/AD	c.488G > A	p.R163H	Het	VUS	Maternal
4	*FLNB*	AR/AD	c.1669C > T	p.P557S	Het	VUS	Paternal
4	*NF1*	AD	c.2991-11C > G	Splicing	Het	VUS	Maternal
5	*SMARCAL1*	AR	c.662G > T	p.R221I	Het	VUS	Maternal
6	*FLNA*	XL	c.2027A > G	p.K676R	Het	VUS	Maternal
8	*TRIP11*	AR	c.4434A > T	p.E1478D	Het	VUS	Maternal
8	*TRIP11*	AR	c.701A > G	p.H234R	Het	VUS	Maternal
8	*COL9A1*	AD	c.432A > G	p.I144M	Het	VUS	Maternal
12	*COL2A1*	AD	c.4393C > T	p.R1465C	Het	VUS	Paternal
12	*HBA2*	AD	c.427 T > C	p.X143Q	Het	VUS	Paternal
13	*PTH1R*	AD/AR	c.629C > T	p.A210V	Het	VUS	Maternal
14	*RPGRIP1L*	AR	c.3272G > A	p.R1091Q	Het	VUS	Paternal
14	*RPGRIP1L*	AR	c.1960G > A	p.E654K	Het	VUS	Paternal

## Data Availability

The data used to support the findings of this study are available from the corresponding author upon request.

## Supplementary Materials

Supplementary Materials Supplementary material of the description of NGS. Supplementary Table S1: 225 genes included in the skeletal gene panel.
